The article "Optimizing the Extraction Conditions of Hydroxytyrosol from Olive Leaves Using a Modified Spherical Activated Carbon: A New Experimental Design" was published in 2022. Journal: Biomed Res Int.

# Optimizing the Extraction Conditions of Hydroxytyrosol from Olive Leaves Using a Modified Spherical Activated Carbon: A New Experimental Design

**DOI:** 10.1155/2022/6199627

**Published:** 2022-05-17

**Authors:** Fatma Hadrich, Sven-Uwe Geißen, Mohamed Chamkha, Sami Sayadi

**Affiliations:** ^1^Environmental Bioprocesses Laboratory, Center of Biotechnology of Sfax, P.O. Box 1177, 3038 Sfax, Tunisia; ^2^Technische Universitat Berlin, Straße des 17. Juni 135, 10623 Berlin, Germany; ^3^Biotechnology Program, Center of Sustainable Development, College of Arts and Sciences, Qatar University, Doha 2713, Qatar

## Abstract

The purification of hydroxytyrosol from olive leaves extract by modified activated carbon was studied experimentally in a batch system and a column by adsorption and desorption processes. The extraction yield reached 90% of hydroxytyrosol, which is the major compound found in the extract. Despite the abundance of research on extracts of hydroxytyrosol from olive leaves, it seems that the applied methods can be further improved. In this study, several approaches were applied to optimize the extraction conditions of this molecule. Hence, the response surface method and the Box-Behnken design (BBD) were used to evaluate the effect of the temperature, time, and adsorbent dose on the hydroxytyrosol recovery. Moreover, adsorption isotherm, kinetics, and thermodynamic studies were also performed to clarify the nature of the process. The main finding was the obtainment of a maximum adsorption yield of 97.5% at an adsorbent/adsorbate ratio of 1 : 20, after a 6 h cycle and at a temperature of 30°C. Furthermore, adsorption process seemed to fit best with Freundlich model. In addition, the thermodynamic study describes a spontaneous and endothermic process. Desorption assay using ethanol helped to recover 73% of hydroxytyrosol. Furthermore, the HPLC analysis of fractions after column adsorption showed a simple peak of hydroxytyrosol with purity higher than 97% and a flavonoids-rich fraction. These findings would indicate that this separation method for the recovery of phenolic compounds with high antioxidant activity can be a very promising one.

## 1. Introduction

Phenolic compounds are secondary metabolites and are widely distributed in plant biomass. These compounds have attractive pharmacological activities such as antioxidant, anticancer, and antidiabetic and are used in the pharmaceutical, cosmetic, and nutritional industries [1].

Unfortunately, an important fraction of these compounds has always been neglected and rejected within solid and liquid byproducts generated from food and agroindustrial processes.

The efficient extraction of polyphenols from waste materials leads to their value-added utilization, with advantages in diverse aspects including environmental, sustainability, and health [2, 3].

The article "Optimizing the Extraction Conditions of Hydroxytyrosol from Olive Leaves Using a Modified Spherical Activated Carbon: A New Experimental Design" was published in 2022. Journal: Biomed Res Int.

Olive leaves (OL) are a considerable byproduct of olive fruit collection and olive oil industry. Şahin and Bilgin [4] revealed that OL contained high contents of polyphenols compared with other food wastes. Indeed, oleuropein is the major phenolic compound, but we found several other flavonoids. In particular, hydroxytyrosol (HT) was obtained after oleuropein hydrolysis or after enzymatic catalysis. This compound presented biological properties that proved to be efficient against diseases such as obesity [5], cancer [6], diabetics [7], and inflammation [8]. For this reason, Abaza et al. (2016) rightly observed that researchers focused on inventing new ways of extracting polyphenols from OL in the last decade [9].

Many procedures including solvent extraction, product separation, and concentration stages were attempted to obtain a phenolic-enriched extract. However, environmental and time-consuming issues caused by these methods compelled researchers to develop simpler, more efficient, and more cost-effective technologies [10]. Therefore, new technologies started suggesting replacements for traditional methods. In this context, adsorption technology offered a simpler and more efficient process appropriate for thermosensitive compounds. This overall process was of great importance and interest since it allowed to simultaneously extract and purify the target compounds and to reduce the number of separation stages [11, 12]. Moreover, this process helped to reduce the degradation of the adsorbate and to avoid the use of toxic solvents [13].

Many researches have shown the efficiency of several adsorbents to remove pollutants including phenols, dye, and pharmaceutical wastes [14–16]. Indeed, researchers have revealed the potential efficiency of graphene oxide and magnetic multiwalled carbon nanotubes-loaded alginate adsorbents to remove dye from textile wastewater [17–19]. Kalash and Albayati have reported the use of mesoporous silica MCM-41 to eliminate polycyclic aromatic hydrocarbons compounds (PAHs) [20]. Similarly, several studies have focused on the adsorption of antibiotics using activated carbon coated by nanoparticles or by mesoporous silica because of the high mechanical stability and large and adjustable pores [21–23]. In fact, activated carbon (AC) was the most popular adsorbent used to remove pollutants from wastewater due to its high adsorption efficiency and the ability of reusability. AC can be produced from various agriculture wastes such as rice husks [24], eucalyptus bark [25], and pomegranate peel [26].

The article "Optimizing the Extraction Conditions of Hydroxytyrosol from Olive Leaves Using a Modified Spherical Activated Carbon: A New Experimental Design" was published in 2022. Journal: Biomed Res Int.

Furthermore, adsorption of natural compounds has attracted a great attention since it leads to the purification and the recovery of high antioxidants compounds which exhibits pharmacological properties. In this context, Datta et al. have reported that polyphenols from ginger rhizomes was purified using anion exchange Amberlite [27]. García-Pérez et al. [28] have explored the adsorption of gallic and polyphenols from *Bryophyllum* extracts using AC. Additionally, it has been reported that tyrosol and hydroxytyrosol was separated from OMW using diverse adsorbents. For example, natural zeolites, dried *Azolla* plant, and Amberlite XAD16 resin were tested for their adsorption capacity [29]. Other adsorbents included the use of graphene oxide which was also explored [30]. To our knowledge, few studies were conducted on the recovery of polyphenols from olive leaves using adsorption process. For this reason, this work purported to develop an integrated method for the separation of polyphenols from olive leaves hydrolyzed extract using modified activated carbon. To attempt these objectives, an optimization step of adsorption variables was evaluated using the response surface methodology (RSM). Moreover, kinetic and thermodynamic parameters were further investigated to explore the interaction mechanism between adsorbent/adsorbate.

## 2. Experimental

### 2.1. Materials and Methods

All reagents and solvents were provided by Bioscience and Sigma-Aldrich. OL samples were collected in the area of Sfax (the South of Tunisia). Dried leaves were powdered and stored in the dark. The extraction was carried out in water at 100°C. The hydrolysis was carried out using 2 M HCl solution (4 : 1 v/v). The extract was filtered to remove any residual solid and then stored at 4°C. The polymer-based activated carbon (AC) was provided by Technische Universitat Berlin (Industrial Product). This adsorbent is efficient for the separation of molecules or pollutants in fluid solutions. The surface area determined by Brunauer-Emmett-Teller (BET) method was measured in SMART SORB 92/93 instrument by using the ASTM Standard Test Method for Carbon Black-Total and External Surface Area by Nitrogen Adsorption (ASTM D6556-04). The surface area was 1736 m^2^/g, and the other parameters were provided in Table 1.

### 2.2. Physicochemical Characterization of Olive Leaves Extract (OLE)

The main characteristics of the tested OLE are reported in Table 2. Total solids were measured by weighing samples before and after drying overnight at 105°C. Volatile solid (VS) was calculated by loss on ignition at 600°C for 2 h. The mineral content was analyzed by flame atomic absorption spectrometry.

The article "Optimizing the Extraction Conditions of Hydroxytyrosol from Olive Leaves Using a Modified Spherical Activated Carbon: A New Experimental Design" was published in 2022. Journal: Biomed Res Int.

The polyphenols concentration in OLE after hydrolysis (OLHE) was quantified according to the modified method described by Singleton et al. [31] using gallic acid as standard.

The identification and the quantification of phenolic compound was monitored using HPLC chromatography at 254, 280, and 320 nm. The separation of the different compounds was performed for an overall 45 min. The flow rate was 0.1 mL min^−1^, and the sample volume injected into HPLC was 20 *μ*L. The gradient elution was employed to separate phenolic compound where the solvents A and B, used as mobile phases, were 0.01% acetic acid in pure water and acetonitrile, respectively.

### 2.3. Adsorption Isotherm Determination

The solution of olive leaves was prepared in molarities in order to make different concentration by adding a constant volume of water for each weight of olive leaves. The adsorbent was added in the second flask by adjusting different mass ratio of 1 : 10, 1 : 15, 1 : 20, 1 : 25, and 1 : 30, and the reactor contents were stirred for different times at 10, 20, and 30°C. Langmuir and Freundlich adsorption isotherm were used to model the equilibrium data for HT adsorption. The equations and parameters related to both models were calculated.

The Langmuir model assumes the formation of monolayer adsorption with equal heat of adsorption on the surface [32]. The equation is determined as follows:

(1) $$\begin{array}{c} \text{qe}=\frac{\text{qm}.\text{KL}.\text{Ce}}{1+\text{KL}.\text{Ce}} \end{array}$$

The Freundlich isotherm characterizes the adsorption on heterogeneous surfaces. The Freundlich equation is described as follows:

(2) $$\begin{array}{c} \text{qe}=\text{Kf}.{\text{Ce}}^{1/\text{n}} \end{array}$$

All parameters related to the adsorption isotherms are determined. The maximum adsorption capacity (qm) and the adsorption coefficient (*K*_*L*_) were measured. Moreover, the values related to the Freundlich model including Freundlich adsorption constants, coefficients, *n*, and *K*_*f*_ were measured.

### 2.4. Adsorption and Desorption Kinetics

Adsorption was carried out under stable conditions at 25°C in a 250-mL Erlenmeyer (200 rpm). Briefly, 100 mL of OLHE was introduced into the flask, and a mass of AC was added.

Then, the mixture was put in shaker at 180 rpm. Samples were taken after defined time intervals of 10, 20, 30, and 60 min and 2, 3, 4, 5, and 6 h. The concentration of the target compound within time was measured. Since the state of equilibrium was not reached after 6 h, the experiment was extended to 12 h and 24 h. After equilibrium was reached, the resin was washed with water. After that, the desorption experiment was carried out with 100 mL of 100% and 70% ethanol for 6 h at 180 rpm. A sample of 1 mL was taken after 10, 20, 30, and 60 min and 2, 3, 4, 5, and 6 h. The HT concentration was measured by HPLC.

The article "Optimizing the Extraction Conditions of Hydroxytyrosol from Olive Leaves Using a Modified Spherical Activated Carbon: A New Experimental Design" was published in 2022. Journal: Biomed Res Int.

The adsorption capacity (qe) of AC at equilibrium (mg/g), the adsorption efficiency *A* (%) and the desorption efficiency *D* (%) were calculated as follows:

(3) $$\begin{array}{c} \text{qe}=\frac{V\left(\text{Co}-\text{Ceq}\right)}{m}, \end{array}$$

where *C*_0_ (mg.L^−1^) and *C*_eq_ (mg.L^−1^) are the initial and the final concentrations of HT, *V* is the volume (L) of sample, and *m* is the adsorbent mass (g).

(4) $$\begin{array}{c} A\left(\%\right)=\frac{\left(\text{Co}-\text{Ceq}\right)}{\text{co}}*100,\\ D\left(\%\right)=\frac{Cd}{\left(Co-Ceq\right)}*100, \end{array}$$

where *C*_*d*_ is the concentration of HT in the desorption solution (mg.mL^−1^).

### 2.5. Experimental Design

Experimental designs are usually for the optimization of the efficacy of independent variables on the process [33]. In this work, response surface methodology (RSM) using Box-Behnken design (BBD) with three factors and three levels was applied to determine the hydroxytyrosol adsorption yield under the optimum operational conditions: temperature (10-30°C), AC:OLHE ratios (0.1–0.3), and adsorption time (1-6 h) (Table 3). The BBD consists of 15 experiments with three replicates of the center point. The influence of the process variables could be represented by a polynomial equation to predict the responses in coded values within the ranges used. Design expert software (trial version 10.0.0) was used to determine the number of errors associated and the values of correlation coefficients (Ma et al., 2014).

The following second-order polynomial equation presents the fitted normalized data.

(5) $$\begin{array}{c} y=a0+\overset{n}{\underset{i=1}{\sum }}aixi+\overset{n}{\underset{i=1}{\sum }}aiix^{2}i+\overset{n-1}{\underset{i=j}{\sum }}\overset{n}{\underset{j=i+1}{\sum }}aijxij, \end{array}$$

where *a*0 is the constant; *ai* is the linear behavior of the model; *aii* is the quadratic coefficient, and *aij* is the coefficient of interaction between two independent variables *xi* and *xj*.

The analysis of variance (ANOVA), describing the integrity of the fitted model on the normalized data, was evaluated by determining the lack of Fit, Fisher *F*-test, and correlation coefficient (*R*^2^ value). The significance of the independent variables and the model was measured by determining the 95% probability test (*p* < 0.05). 3D plots of the model were plotted to depict the interaction between process variables and the predicted response.

### 2.6. Column Test

Column test was performed using a water-jacketed glass column with a diameter of 1.6 cm and a length of 23 cm with repeated adsorption and desorption cycles. The column was preconditioned by adding water. During the adsorption cycle, the OLHE solution was continuously loaded into the column with an adjusted flow rate of 1.2 mL.min^−1^ controlled by a metering pump until the column saturation. The concentration of hydroxytyrosol and phenolic compounds was controlled by HPLC. After column saturation, the fractions were recuperated after washing the column by water and then with EtOH until the concentration of HT reached the 0.007 mg. mL^−1^. The saturated column was regenerated with an optimized regeneration solution (0.5 M NaOH) and then rinsed with deionized water for the next adsorption cycle. The column adsorption capacity in each cycle was calculated.

The article "Optimizing the Extraction Conditions of Hydroxytyrosol from Olive Leaves Using a Modified Spherical Activated Carbon: A New Experimental Design" was published in 2022. Journal: Biomed Res Int.

## 3. Results and Discussion

### 3.1. OLE Hydrolyzed Extract Composition

Table 4 shows the mineral content of OLE hydrolysis after incineration. The data clearly revealed that this extract was a rich source of minerals. Indeed, calcium was the predominant element (624.0 mg/100 g dry matter) present in the extract, followed by potassium (336 g/100 g). These findings support the previous results by Bahloul et al. [34] who showed that the calcium was the predominant mineral in different varieties of OL and that its amounts ranged between 600 mg/100 g and 982 mg/100 mg. Similarly, Saidana et al. [35] showed that the accumulation of the calcium minimized the level of Na. Additionally, Bustan et al. [36] have reported that in arid environment, tolerable concentrations of Ca are acceptable in olive to protect against Na toxicity. Moreover, as was reported in previous works, phosphorus was found OTLE at 125 mg/100 g [37]. These scholars explained that because phosphorus was an essential macroelement, it was not commonly applied in olive tree plantations. Consequently, they induced that this vegetable material could contribute to the maintenance of appropriate levels of nutriments for the human body. Similarly, El and Karakaya [38] revealed that hydrolysis increased the polyphenol concentration in OLE. These scholars explained that this increase in concentration characterized OLE by a strong radical scavenging effect. In fact, oleuropein and hydroxytyrosol have the same antioxidant activity with vitamins C and E [4].

### 3.2. Isotherm Adsorption

Figure 1(a) shows the Langmuir adsorption model of HT on a homogenous surface at different temperatures. As can be seen in this graphic presentation, there was a monolayer adsorption on a homogenous surface with the same affinity in all the adsorption sites with a negligible interaction between the adjacent adsorbed molecules.

The article "Optimizing the Extraction Conditions of Hydroxytyrosol from Olive Leaves Using a Modified Spherical Activated Carbon: A New Experimental Design" was published in 2022. Journal: Biomed Res Int.

The correlation coefficient *R*^2^ was used to determine the closest data percent values to the line of the best fit. The first observation was that a simple comparison of regression coefficient (*R*^2^) would reveal that experimental data fitted better the Freundlich model (Figure 1(b)). This would imply that the contact surface between the adsorbent and adsorbate was heterogeneous.  Table 5 shows all parameters related to the adsorption isotherms. The maximum adsorption capacity (qm) and the adsorption coefficient (*K*_*L*_) were measured. Moreover. All the Freundlich adsorption constants, coefficients, *n*, and *K*_*f*_ were resumed in Table 5. The second observation would be related to the 1/*n* value calculated for this model. This value ranged between 0 and 1, signifying a favorable physical adsorption process and, therefore, suggesting a monolayer adsorption according to the IUPAC indication.

The third observation was that the *K*_*f*_ values increased with the increase of temperature, implying that this adsorption process was endothermic. This finding confirmed many previous works on the extraction of different plant extracts. For example, it supported Ribeiro et al.'s [39] observation that Langmuir and Freundlich models were perfectly fit to establish the adsorption equilibrium data of plant extracts.

Equally, this work was in agreement with García Pérez et al. [28] who demonstrated that both Langmuir and Freundlich isotherm models fitted the equilibrium data of the adsorption process of gallic acid and propyl gallate. Similarly, this study was in line with Lehmann et al. [40] who revealed that the Langmuir model fitted the recovery of polyphenolic compounds from Switchgrass extract. Ena et al. [41] have reported that the Freundlich model was predicted the experimental data on recovery of HT from olive mill wastewater by adsorption on granular activated carbon. In contrary, Aliakbarian et al. showed that Langmuir isotherm Langmuir model fitted better for the adsorption of phenolic compounds from olive mill wastewater (OMW) [42].

Furthermore, to get more information on the adsorption mechanism including surface interactions and diffusion within the pores, this study applied the kinetic model investigation. Therefore, following Kadhum et al. [43], the pseudo-first-order and pseudo-second-order models and intraparticle were used to describe HT adsorption on AC.

As can be seen in Table 5, *R*^2^ values indicated that the pseudo-second-order model fitted very well the adsorption of HT on AC. Moreover, the pseudo-second-order kinetic model operated under the assumption that the adsorption concentration of adsorbate was closely related to the rate-limiting step in the adsorption process.

The article "Optimizing the Extraction Conditions of Hydroxytyrosol from Olive Leaves Using a Modified Spherical Activated Carbon: A New Experimental Design" was published in 2022. Journal: Biomed Res Int.

### 3.3. Adsorption and Desorption Kinetics

Figure 2 illustrates the adsorption kinetics in a batch system. As can be seen in Figure 2(a), within the first 30 min, there was an adsorption of 65% of HT into AC. However, after 5 h, the adsorption yield reached 96.85%. After 24 h, adsorption seemed to stabilize at 98.5%.

Therefore, for reasons of cost-effectiveness, this study would recommend an adsorption time of six hours especially that adsorption at this time would yield 97.5% of HT adsorption. The addition of only 1% in 18 hours would be considered unproductive. Our finding showed that the novel adsorbent used in this study seem to be more efficient than Azolla, XAD16, IRAD 96, and XAD7 which showed an adsorption rate of 97.53% [44–48]. It has been reported that TRI-SBA15 exhibits slightly higher adsorption efficiency of tyrosol [49]. This result proved that adsorbents based with activated carbon showed the best uptake of phenolic compounds.  Table 6 summarizes the recovery percentage of HT using different adsorbents. Firstly, Figure 1(b) shows the desorption kinetic conducted with 100% and 70% ethanol over a period of 24 h. The recovery yields for HT after sequential desorption with both solvents revealed no significant differences. However, desorption with 100% ethanol seemed to be more appropriate because it reduced the concentration of salt and carbohydrates.

This finding confirms Zagklis et al.'s [45] recommendation to prewash the loaded adsorbent with deionized water prior to the desorption with ethanol to reduce the interfering matrix on the adsorbent and to elute carbohydrates. Additionally, these scholars revealed that the subsequent application of ethanol after deionized water increased the concentration of HT in the desorption solution because of a lesser competitive elution with sugars.

Secondly, Figure 2(b) shows that during sequential desorption, the desorption yield increased linearly to 40% after 90 min. This yield continued its sharp increase until reaching 73% after 5 h. Then, the desorption seemed to stabilize for the rest of the 24 hours. Therefore, this work would consider the period of 5 h as the optimum desorption time.

### 3.4. Optimization of Process Parameters

The aim of this experiment was to find the optimum of values for the operating conditions that would enhance the efficiency of HT adsorption. The regression analysis resulted in a second order polynomial equation that would help to compute the predicted responses of HT adsorption in terms of coded variables

(6) $$\begin{array}{c} Y=96.85+14.81\;A+2.07\;B+9.63\;C-5.16\;AC–9.59\;A^{2}-4.26\;B^{2}-7.62\;C^{2}. \end{array}$$

where *Y* is the adsorption percentage of HT; *A* is the ratio adsorbent-adsorbate; *B* is the temperature; *C* is the time; AC is the interaction factor; and *A*^2^, *B*^2^, and *C*^2^ are the quadratic terms included.

The article "Optimizing the Extraction Conditions of Hydroxytyrosol from Olive Leaves Using a Modified Spherical Activated Carbon: A New Experimental Design" was published in 2022. Journal: Biomed Res Int.

#### 3.4.1. Analysis of the Variance (ANOVA)

The ANOVA results of the fitted quadratic model are presented in Table 7. The model *F*-value was 70.33 implying that the model was significant (*p* < 0.0001). The adequate precision ratio was equal to 27.961; so >4 and indicating an adequate signal. Moreover, the value of *R*^2^ and the adjusted determination coefficient (*R*^2^ adj) indicating the goodness of fit of the regression procedure undertaken were 0.992 and 0.978, respectively. As can be seen in Table 7, *A*, *B*, *C*, AC, *A*^2^, *B*^2^, and *C*^2^ are the significant model terms having an F-statistics probability value of less than 0.05. Based on 2D, the adsorbent-adsorbate ratio and the time had the most significant impact on the model. Moreover, Figure 3 shows the correlation between actual values and predicted values for the yield of HT adsorption. The scattering of the data points along the diagonal line seemed to confirm the goodness fit of the model.

#### 3.4.2. Optimization of HT Adsorption

Figure 4 shows that the time and the ratio of adsorbent-adsorbate had the most significant influence on the adsorption yield. Firstly, Figure 4(a) shows that the time increased the adsorption efficacy until the equilibrium was reached. Consequently, the maximum HT adsorption was reached after 4 hours.

This can be explained by the fact that the adsorption process was fast in the beginning of the process because of the availability of the active sites at the contact area. However, the longer the process was, the more saturated the adsorbent surface became because of the molecule binding into receptors. Secondly, a ratio of 1 : 20 seemed to be the most appropriate since the HT adsorption yield reached 97% at this value. In addition, the use of the ratio 1 : 30 seemed to have increased the adsorbent mass. Still worse, a ratio of 1 : 40 did not improve the adsorption performance. This result can be explained by the bending of most molecules of the adsorbate. This finding was consistent with Yangui et al.'s results [31]. These scholars reported that the increase in adsorbent concentration (more than 50 g. L^−1^) did not enhance the adsorption efficiency. They explained this by the aggregation and the agglomeration of the adsorbent particles which caused a decrease in total surface area of the adsorbent.

Figures 4(b) and 4(c) illustrate the effect of temperature on the adsorption yield. It seemed that there was little effect of this variable on HT adsorption. Indeed, the adsorption capacity after 6 h was 0.0697, 0.0293, and 0.0213 at 10, 20, and 30°C, respectively.

The article "Optimizing the Extraction Conditions of Hydroxytyrosol from Olive Leaves Using a Modified Spherical Activated Carbon: A New Experimental Design" was published in 2022. Journal: Biomed Res Int.

### 3.5. Thermodynamic Study of Adsorption

Table 8 shows the effect of temperature on the adsorption of OLHE. The influence of the temperature on the adsorption of OLHE was explored, and the result was shown in Table 8. The thermodynamics parameters such as enthalpy change (∆*H*, kJ/mol), free energy change (∆*G*, kJ/mol), and entropy change (∆*S*, kJ/mol K) were estimated using the following equations [32].

(7) $$\begin{array}{c} \Delta r\;G\circ =-\text{R}.\text{T}.\text{LnKc}\\ \text{Ln Kc}=\frac{∆S\;}{R}-\frac{∆H}{RT} \end{array}$$

The Δ*H* and Δ*S* values were measured from the slope and the intercept of the linear correlation between Ln (Kc) and 1/T known as the Van't Hoff plot. *R* is the ideal gas constant (8.314 J K^−1^ mol^−1^), and *T* is the temperature in Kelvin (K).

Firstly, the positive values of ∆*H* confirmed the endothermic nature of the adsorption process. This finding, confirms Yangui et al.' s [31] observation about the endothermic nature of the adsorption process of polyphenols contained in olive mill wastewater (OMW) at temperatures ranging between 20°C and 40°C. Additionally, this study totally agrees with a previous explanation provided by García-Araya et al. [50] and Singh et al. [51] when they tested the use of endothermic processes for the adsorption of phenolic compounds on AC. These scholars discovered that within this process the increase of temperature led to a better diffusion of the adsorbate in the microporous structure. Therefore, they proposed the plausible explanation of the existence of temperature dependent electrostatic interactions and dispersion forces in the process.

Secondly, the value of ∆*H* was < 40 kJ/mol. This would indicate that the dominating mechanism was a physical adsorption as was demonstrated in a previous work by Gao et al. [52].

Thirdly, the negative value of Gibbs energy (∆*G*) suggested that the adsorption of polyphenols was a spontaneous process. Nevertheless, the absolute values of ∆*G* confirmed that the adsorption phenomenon would occur at a higher temperature since increasing the temperature increased the value of ∆*G*. This result was consistent with the adsorption equilibrium study conducted by Ding et al. [53]. These scholars demonstrated that the absolute value of ∆*G* was < 20 KJ/mol indicating that the adsorption of OTLHE onto AC occurred via physical adsorption.

Finally, Table 8 shows that the entropy change (∆*S*) had a positive value. This would imply that this parameter plays a contributing role in reflecting whether the organization of adsorbate molecules into adsorbate/adsorbent interface became random. The randomness of solute adsorption increased at the solid–liquid interface. This phenomenon was probably due to the water molecules desorption previously adsorbed onto the AC.

The article "Optimizing the Extraction Conditions of Hydroxytyrosol from Olive Leaves Using a Modified Spherical Activated Carbon: A New Experimental Design" was published in 2022. Journal: Biomed Res Int.

### 3.6. Adsorption of Phenolic Compounds in Column

The data obtained from the batch were confirmed in column test. In fact, our findings revealed that 80% of hydroxytyrosol was retained. The identification of the polyphenols in OLHE before adsorption exhibit the hydroxytyrosol as a major compound, and we note the presence of other flavonoids (Figure 5(a)). After desorption, the chromatogram of fractions showed a monomodal pic of hydroxytyrosol, with a purity degree higher than 97% (Figure 5(b)). This result is in accordance with our previous research [54], in which we have demonstrated the purification of hydroxytyrosol using semipreparative HPLC. Moreover, flavonoids rich-fraction was obtained. The effect of flow rate was discussed according to the breakthrough curve obtained using different flow rates at 1.2 and 2.5 mL/min (data not shown). Our results showed that at high flow rate, the front of the adsorption zone quickly reached the top of the column and consequently lead to the early saturation and less adsorption uptake. Lower flow rate has resulted in longer contact time as well as shallow adsorption zone.

The stability of the process was evaluated by the reuse of the adsorbent for novel cycles. The recyclability was evaluated as follow. After the first cycle of adsorption and desorption, the activated carbon was regenerated twice with NaOH (0.5 M) and then was rinsed several times with ultrapure water. The adsorbent was placed subsequently in the incubator at 50°C. After that, the resin was extracted with NaOH (1 M) and washed with deionized water before drying in the oven at 105°C for 1 h. The regenerated adsorbent was used later for a new adsorption. Our outcomes revealed that adsorption and desorption capacities were found to be 81.4 ± 0.9% and 70.2 ± 3.1%, respectively.

## 4. Conclusion

The present study attempted to explore ways of optimizing the extraction conditions of HT adsorption from OL using modified AC. The main finding was the obtainment of a maximum adsorption yield of 97.53% at an adsorbent/adsorbate ratio of 1 : 20, after a 6 h cycle and at a temperature of 30°C. Freundlich model was found to be suitable for a monolayer adsorption, and an endothermic reaction was occurred. The column experiment revealed that a flavonoid-rich fraction was obtained, and additional investigations were applied to recover and purify other compounds found in the extract. This improved method would provide an environmentally friendly approach for the recovery of high-value molecules which can be used in pharmaceutical and cosmetic industries.

The article "Optimizing the Extraction Conditions of Hydroxytyrosol from Olive Leaves Using a Modified Spherical Activated Carbon: A New Experimental Design" was published in 2022. Journal: Biomed Res Int.

## Figures and Tables

**Figure 1:** Langmuir (a) and Freundlich (b) isotherm adsorption models at 10, 20, and 30°C. qe = adsorption capacity; Ce = equilibrium HT concentration.

**Figure 2:** Adsorption efficiency (*A*%) (a) and desorption percentage (*D*%) (b) of HT from olive leaves extract using modified activated carbon (AC).

**Figure 3:** Correlation of the actual experimental and the models predicted values for the yield HT adsorption.

**Figure 4:** 3D plots of the effect of the interactions between HT adsorption variables: (a) adsorbent concentration and time, (b) temperature and time, and (c) adsorbent concentration and temperature.

**Figure 5:** HPLC chromatograms of raw olive leaves extract (a) and extract after adsorption into activated carbon (b).

**Table 1:** Characteristics of activated carbon.

Characteristics	Adsorbent
Granulometry	(>80%) 0.315-0.58 mm
Specific surface area	1736 m^2^/g
Total ashes (%)	0.2%
Moisture	0.1%
Particle size	0.457 mm
Apparent density	489 kg/m^3^
Abrasion strength	98.6%

**Table 2:** Main characteristics of olive leaves extract after hydrolysis.

Polyphenols (mg/mL)	18.36 GAE
Total solid (%)	15.33
Mineral content (%)	34.66
Volatile solids(%)	50

**Table 3:** Box-Behnken experimental design with three variables (*A*, *B*, and *C*) and the yield adsorption of hydroxytyrosol on AC (*Y*).

	Adsorbent ration	Temperature	Time	HT adsorption (%)
Test	*A*	*B*	*C*	*Y*
1	01 : 10	10	3.5	70.77
2	01 : 30	10	3.5	95.98
3	01 : 10	30	3.5	68.33
4	01 : 30	30	3.5	99.01
5	01 : 10	20	1	49,42
6	01 : 30	20	1	91.37
7	01 : 10	20	6	78.61
8	01 : 30	20	6	98.54
9	01 : 20	10	1	70.41
10	01 : 20	30	1	79.88
11	01 : 20	10	6	92.25
12	01 : 20	30	6	97.53
13	01 : 20	20	3.5	96.85
14	01 : 20	20	3.5	96.85
15	01 : 20	20	3.5	96.85

**Table 4:** Minerals composition of olive leaves extract after hydrolysis (mg.g^−1^ dry matter).

Minerals	Concentration (mg/100 g)
Fe	30
Na	12
K	336
Ca	624
Zn	ND
Mn	ND
Cu	ND

**Table 5:** Adsorption isotherms and kinetic models of HT adsorption.

Models	Equations	Constants		
Langmuir	$qe=\frac{qmKl.Ce}{1.Kl.Ce}$	*K*_*L*_ (L.g^−1^)	*q*_*m*_ (mg.g^−1^)	*R* ^2^
		109.00	91.743	0.998
Freundlich	qe = *k*_*F*_ · *C*_*e*_^1/*n*^	*K*_*F*_ (mg.g^−1^)	*n*	*R* ^2^
		148.41	4	0.996
Pseudo-first-order	$\frac{dq}{dt}=K_{1}.\left(q_{e}‐q_{1}\right)$	*q*_(*e*, calc)_ (mg.g^−1^)	*K*_1_	*R*_1_^2^
		28.18	0.0021	0.96
Pseudo-second-order	$\frac{dq}{dt}=K_{2}.\left(q_{e}‐q_{2}\right)$	*q*_(*e*, calc)_ (mg.g^−1^)	*K*_2_	*R*_2_^2^
		46.3	0.0005	0.9977
Intraparticle diffusion	*q*_*t*_ = *K*_*id*_*t*_1/2_	*K*_*id*_ (mg g^−1^ min^−0.5^)		*R* ^2^
		2.701		0.98

*q*_*e*_: the maximum adsorption capacity (mg g^−1^); *q*_*m*_: the quantity of polyphenols at saturation of monolayer capacity (mg g^−1^); *K*_*L*_: the Langmuir constant; *K*_*F*_: the Freundlich constant; *n*: the Freundlich exponent. *K*_1_: the pseudo-first-order rate constant for adsorption (min^−1^); *K*_2_: the pseudo-second-order rate constant for adsorption (mg. g^−1^ min^−1^); Kid: the rate constant for intraparticle diffusion (mg. g^−1^ min^−0.5^).

The article "Optimizing the Extraction Conditions of Hydroxytyrosol from Olive Leaves Using a Modified Spherical Activated Carbon: A New Experimental Design" was published in 2022. Journal: Biomed Res Int.

**Table 6:** Comparison of several adsorbents efficiency for hydroxytyrosol recovery.

References	Recovery Yield	Adsorbent
Scoma et al. [44]	Removal of 60% phenolic compounds	Amberlite XAD16
Ena et al.[41]	60% of phenolic compounds were adsorbed	Dry Azolla
Zagklis et al. [45]	74% of hydroxytyrosol was recovered	Non ionic XAD4, XAD16 resin
Kaleh et al. [46]	79% of hydroxytyrosol and 95 % of tyrosol were adsorbed	Molecular imprinted polymer
Liu et al. [47]	88.58% of hydroxytyrosol	BMKX-4
Ortega et al. [48]	Amberlyst A26: 98%; Amberlite IRA-67: 57%	Ion-exchange resins: Amberlyst A26 and Amberlite IRA-67
Yangui et al. [49]	91% of Hydroxytyrosol was recovered	TRI-SBA-15

**Table 7:** Analysis of variance of the quadratic model in Box-Behnken design.

Source	Sum of squares	df	Mean square	*F*-value	*p*-value	
Model	3201,44	9	355,72	70,33	< 0.0001	Significant
A (adsorbent ratio)	1755,58	1	1755,58	347,10	< 0.0001	
B (temperature)	34,24	1	34,24	6,77	0,0481	
C (time)	741,51	1	741,51	146,60	< 0.0001	
AB	9,00	1	9,00	1,78	0,2398	
AC	106,61	1	106,61	21,08	0,0059	
BC	4,82	1	4,82	0,9526	0,3739	
*A* ^2^	339,40	1	339,40	67,10	0,0004	
*B* ^2^	67,09	1	67,09	13,26	0,0149	
*C* ^2^	214,39	1	214,39	42,39	0,0013	
Residual	25,29	5	5,06			
Lack of fit	25,29	3	8,43			
Pure error	0,0000	2	0,0000			
Cor Total	3226,73	14				

**Table 8:** Thermodynamic values for HT adsorption onto activated carbon.

Temperature (*K*)	*K*_*c*_ (L.mg^−1^)	∆*H* (kJ.mol^−1^)	∆*S* (kJ.mol^−1^)	∆*G* (kJ.mol^−1^)
283	834,2	36074,446	183,7394	-15834,8521
293	1643,98			-18047,5328
303	2284,91			-19492,9044

## Data Availability

The datasets used and/or analyzed during the current study are available from the corresponding authors on reasonable request.

## References

[1] Szewczyk K., Zidorn C., Biernasiuk A., Komsta Ł., Granica S. (2016). Polyphenols from Impatiens (Balsaminaceae) and their antioxidant and antimicrobial activities. *Industrial Crops and Products*.

[2] Pinelli D., Bacca A. E. M., Kaushik A. (2016). Batch and continuous flow adsorption of phenolic compounds from olive mill wastewater: a comparison between nonionic and ion exchange resins. https://www.hindawi.com/journals/ijce/2016/9349627/.

The article "Optimizing the Extraction Conditions of Hydroxytyrosol from Olive Leaves Using a Modified Spherical Activated Carbon: A New Experimental Design" was published in 2022. Journal: Biomed Res Int.

[3] Fava G., Di Mauro M. D., Spampinato M. (2017). Hydroxytyrosol recovery from olive mill wastewater: process optimization and development of a pilot plant. *CLEAN-Soil, Air, Water*.

[4] Şahin S., Bilgin M. (2018). Olive tree (*Olea europaea* L.) leaf as a waste by-product of table olive and olive oil industry: a review. *Journal of the Science of Food and Agriculture*.

[5] Hadrich F., Mahmoudi A., Bouallagui Z. (2016). Evaluation of hypocholesterolemic effect of oleuropein in cholesterol-fed rats. *Chemico-Biological Interactions*.

[6] De Marino S., Festa C., Zollo F. (2014). Antioxidant activity and chemical components as potential anticancer agents in the olive leaf (Olea europaea L. cv Leccino.) decoction. *Anti-Cancer Agents in Medicinal Chemistry*.

[7] Hadrich F., Garcia M., Maalej A. (2016). Oleuropein activated AMPK and induced insulin sensitivity in C2C12 muscle cells. *Life Sciences*.

[8] Jemai H., Mahmoudi A., Feryeni A. (2020). Hepatoprotective effect of oleuropein-rich extract from olive leaves against cadmium-induced toxicity in mice. *BioMed Research International*.

[9] Abaza L., Taamalli A., Nsir H., Zarrouk M. (2015). Olive tree (Olea europeae L.) leaves: importance and advances in the analysis of phenolic compounds. *Antioxidants*.

[10] Tsao R., Deng Z. (2004). Separation procedures for naturally occurring antioxidant phytochemicals. *Journal of Chromatography B*.

[11] Díaz-Reinoso B., González-López N., Moure A., Domínguez H., Parajó J. C. (2010). Recovery of antioxidants from industrial waste liquors using membranes and polymeric resins. *Journal of Food Engineering*.

[12] Kammerer D. R., Kammerer J., Valet R., Carle R. (2014). Recovery of polyphenols from the by-products of plant food processing and application as valuable food ingredients. *Food Research International*.

[13] Soto M. L., Moure A., Domínguez H., Parajó J. C. (2011). Recovery, concentration and purification of phenolic compounds by adsorption: a review. *Journal of Food Engineering*.

[14] Mukherjee S., Kumar S., Misra A. K., Fan M. (2007). Removal of phenols from water environment by activated carbon, bagasse ash and wood charcoal. *Chemical Engineering Journal*.

[15] Thue P. S., Adebayo M. A., Lima E. C. (2016). Preparation, characterization and application of microwave-assisted activated carbons from wood chips for removal of phenol from aqueous solution. *Journal of Molecular Liquids*.

[16] Pasalari H., Ghaffari H. R., Mahvi A. H., Pourshabanian M., Azari A. (2017). Activated carbon derived from date stone as natural adsorbent for phenol removal from aqueous solution. *Desalination and Water Treatment*.

The article "Optimizing the Extraction Conditions of Hydroxytyrosol from Olive Leaves Using a Modified Spherical Activated Carbon: A New Experimental Design" was published in 2022. Journal: Biomed Res Int.

[17] Azari A., Nabizadeh R., Mahvi A. H., Nasseri S. (2021). Magnetic multi-walled carbon nanotubes-loaded alginate for treatment of industrial dye manufacturing effluent: adsorption modelling and process optimisation by central composite face-central design. *International Journal of Environmental Analytical Chemistry*.

[18] Azari A., Nabizadeh R., Mahvi A. H., Nasseri S. (2020). Integrated fuzzy AHP-TOPSIS for selecting the best color removal process using carbon-based adsorbent materials: multi-criteria decision making vs. systematic review approaches and modeling of textile wastewater treatment in real conditions. *International Journal of Environmental Analytical Chemistry*.

[19] Azari A., Noorisepehr M., Dehganifard E. (2019). Experimental design, modeling and mechanism of cationic dyes biosorption on to magnetic chitosan-lutaraldehyde composite. *International Journal of Biological Macromolecules*.

[20] Kalash K. R., Albayati T. M. (2021). Remediation of oil refinery wastewater implementing functionalized mesoporous materials MCM-41 in batch and continuous adsorption process.

[21] Rashtbari Y., Hazrati S., Azari A., Afshin S., Fazlzadeh M., Vosoughi M. (2020). A novel, eco-friendly and green synthesis of PPAC-ZnO and PPAC-nZVI nanocomposite using pomegranate peel: cephalexin adsorption experiments, mechanisms, isotherms and kinetics. *Advanced Powder Technology*.

[22] Alkafajy A. M., Albayati T. M. (2020). High performance of magnetic mesoporous modification for loading and release of meloxicam in drug delivery implementation. *Materials Today Communications*.

[23] Mahmoudian M. H., Fazlzadeh M., Niari M. H., Azari A., Lima E. C. (2020). A novel silica supported chitosan/glutaraldehyde as an efficient sorbent in solid phase extraction coupling with HPLC for the determination of Penicillin G from water and wastewater samples. *Arabian Journal of Chemistry*.

[24] Balarak D., Mostafapour F. K., Lee S. M., Jeon C. (2019). Adsorption of bisphenol A using dried rice husk: equilibrium, kinetic and thermodynamic studies. *Applied Chemistry for Engineering*.

[25] Zazouli M. A., Azari A., Dehghan S., Malekkolae R. S. (2016). Adsorption of methylene blue from aqueous solution onto activated carbons developed from eucalyptus bark and Crataegus oxyacantha core. *Water Science and Technology*.

[26] Ali I., Afshinb S., Poureshgh Y. (2020). Green preparation of activated carbon from pomegranate peel coated with zero-valent iron nanoparticles (nZVI) and isotherm and kinetic studies of amoxicillin removal in water. *Environmental Science and Pollution Research*.

[27] Datta C., Dutta A., Dutta D., Chaudhuri S. (2011). Adsorption of polyphenols from ginger rhizomes on an anion exchange resin Amberlite IR-400 - study on effect of pH and temperature. *Procedia Food Science*.

The article "Optimizing the Extraction Conditions of Hydroxytyrosol from Olive Leaves Using a Modified Spherical Activated Carbon: A New Experimental Design" was published in 2022. Journal: Biomed Res Int.

[28] García-Pérez P., Losada-Barreiro S., Gallego P. P., Bravo-Díaz C. (2019). Adsorption of gallic acid, propyl gallate and polyphenols from Bryophyllum extracts on activated carbon. *Scientific Reports*.

[29] Padovani G., Pintucci C., Carlozzi P. (2013). Dephenolization of stored olive-mill wastewater, using four different adsorbing matrices to attain a low-cost feedstock for hydrogen photo-production. *Bioresource Technology*.

[30] Şahin S., Ciğeroğlu Z., Özdemir O. K., Elhussein E., Gülmez Ö. (2020). Investigation of graphene oxide as highly selective adsorbent in recovery of hydroxytyrosol from olive mill wastewater. *International journal of Environmental Science and Technology*.

[31] Singleton V. L., Orthofer R., Lamuela-Raventós R. M. (1999). *Oxidants and Antioxidants Part a*.

[32] Alardhi S. M., Alrubaye J. M., Albayati T. M. Adsorption of methyl green dye onto MCM-41: equilibrium, kinetics and thermodynamic studies. https://www.deswater.com/DWT_articles/vol_179_papers/179_2020_323.pdf.

[33] Pizarro C., Sáenz-González C., Pérez-del-Notario N., González-Sáiz J. M. (2012). Development of an ultrasound-assisted emulsification-microextraction method for the determination of the main compounds causing cork taint in wines. *Journal of Chromatography A*.

[34] Bahloul N., Kechaou N., Mihoubi N. B. (2014). Comparative investigation of minerals, chlorophylls contents, fatty acid composition and thermal profiles of olive leaves (Olea europeae L.) as by-product. *Grasas y Aceites*.

[35] Naija D. S., Boussaadia O., Ben Dhiab A., Ben Mariem F., Braham M. (2014). Valorization of the olive sector effluents as potential fertilizers and their impact on biological, physical and chemical properties of the soil. *Research Journal of Agriculture and Environmental Management*.

[36] Bustan A., Avni A., Yermiyahu U. (2013). Interactions between fruit load and macroelement concentrations in fertigated olive (Olea europaea L.) trees under arid saline conditions. *Scientia Horticulturae*.

[37] Cavalheiro C. V., Picoloto R. S., Cichoski A. J. (2015). Olive leaves offer more than phenolic compounds - fatty acids and mineral composition of varieties from Southern Brazil. *Industrial Crops and Products*.

[38] El S. N., Karakaya S. (2009). Olive tree (Olea europaea) leaves: potential beneficial effects on human health. *Nutrition Reviews*.

[39] Ribeiro M. H. L., Silveira D., Ferreira-Dias S. (2002). Selective adsorption of limonin and naringin from orange juice to natural and synthetic adsorbents. *European Food Research and Technology*.

[40] Lehmann M. L., Counce R. M., Counce R. W., Watson J. S., Labbé N., Tao J. (2018). Recovery of phenolic compounds from switchgrass extract. *ACS Sustainable Chemistry and Engineering*.

The article "Optimizing the Extraction Conditions of Hydroxytyrosol from Olive Leaves Using a Modified Spherical Activated Carbon: A New Experimental Design" was published in 2022. Journal: Biomed Res Int.

[41] Ena A., Pintucci C., Carlozzi P. (2012). The recovery of polyphenols from olive mill waste using two adsorbing vegetable matrices. *Journal of Biotechnology*.

[42] Aliakbarian B., Casazza A. A., Perego P. (2015). Kinetic and isotherm modelling of the adsorption of phenolic compounds from olive mill wastewater onto activated carbon. *Food Technology and Biotechnology*.

[43] Kadhum S. T., Alkindi G. Y., Albayati T. M. (2021). Eco friendly adsorbents for removal of phenol from aqueous solution employing nanoparticle zero-valent iron synthesized from modified green tea bio-waste and supported on silty clay. *Chinese Journal of Chemical Engineering*.

[44] Scoma A., Bertin L., Zanaroli G., Fraraccio S., Fava F. (2011). A physicochemical-biotechnological approach for an integrated valorization of olive mill wastewater. *Bioresource Technology*.

[45] Zagklis D. P., Vavouraki A. I., Kornaros M. E., Paraskeva C. A. (2015). Purification of olive mill wastewater phenols through membrane filtration and resin adsorption/desorption. *Journal of Hazardous Materials*.

[46] Kaleh Z., Geißen S. U. (2016). Selective isolation of valuable biophenols from olive mill wastewater. *Journal of Environmental Chemical Engineering*.

[47] Liu B., Liu J., Huang D., Pei D., di D. (2020). Separation and purification of hydroxytysol and oleuropein from Olea europaea L. (olive) leaves using macroporous resins and a novel solvent system. *Journal of Separation Science*.

[48] Víctor-Ortega M. D., Ochando-Pulido J. M., Martínez-Ferez A. (2016). Performance and modeling of continuous ion exchange processes for phenols recovery from olive mill wastewater. *Process Safety and Environmental Protection*.

[49] Yangui A., Abderrabba M., Sayari A. (2017). Amine-modified mesoporous silica for quantitative adsorption and release of hydroxytyrosol and other phenolic compounds from olive mill wastewater. *Journal of the Taiwan Institute of Chemical Engineers*.

[50] García-Araya J. F., Beltrán F. J., Álvarez P., Masa F. J. (2003). Activated carbon adsorption of some phenolic compounds present in agroindustrial wastewater. *Adsorption*.

[51] Singh K. P., Malik A., Sinha S., Ojha P. (2008). Liquid-phase adsorption of phenols using activated carbons derived from agricultural waste material. *Journal of Hazardous Materials*.

[52] Gao Z. P., Yu Z. F., Yue T. L., Quek S. Y. (2013). Adsorption isotherm, thermodynamics and kinetics studies of polyphenols separation from kiwifruit juice using adsorbent resin. *Journal of Food Engineering*.

The article "Optimizing the Extraction Conditions of Hydroxytyrosol from Olive Leaves Using a Modified Spherical Activated Carbon: A New Experimental Design" was published in 2022. Journal: Biomed Res Int.

[53] Ding L., Deng H., Wu C., Han X. (2012). Affecting factors, equilibrium, kinetics and thermodynamics of bromide removal from aqueous solutions by MIEX resin. *Chemical Engineering Journal*.

[54] Hadrich F., Bouallagui Z., Junkyu H., Isoda H., Sayadi S. (2015). The *α*-glucosidase and *α*-amylase enzyme inhibitory of hydroxytyrosol and oleuropein. *Journal of Oleo Science*.

